The article "Effect of Programmed Nursing Plan Based on Thinking Map Guidance Mode on Hemodynamics and Intestinal Function Recovery of Patients Undergoing Endoscopic Retrograde Cholangiopancreatography" was published in 2022. Journal: Emerg Med Int.

# Effect of Programmed Nursing Plan Based on Thinking Map Guidance Mode on Hemodynamics and Intestinal Function Recovery of Patients Undergoing Endoscopic Retrograde Cholangiopancreatography

**DOI:** 10.1155/2022/6555150

**Published:** 2022-05-14

**Authors:** Yan Lu, Feifei Wang

**Affiliations:** Department of Gastroenterology, Huzhou Central Hospital& Central Hospital, affiliated to Huzhou Teachers College, Huzhou, Zhejiang 313000, China

## Abstract

ERCP is an effective method for the diagnosis and treatment of pancreatic and biliary diseases. With the improvement of endoscopes by researchers and the intubation and angiography technologies of medical workers, the role of ERCP in the diagnosis and treatment of pancreatic and biliary diseases has become increasingly important. Although ERCP is a minimally invasive diagnostic technique, it still falls into the category of surgery, and thus the physical and psychological dysfunction of patients undergoing ERCP caused by various factors such as surgery cannot be ignored. This study explored the effects of the procedural nursing plan based on the thinking map guidance mode on hemodynamics and intestinal function recovery of ERCP patients. The results showed that this plan could reduce the effects of ERCP on hemodynamics of patients, promote intestinal function recovery, relieve their bad psychology, reduce postoperative complications, and help to improve patients' satisfaction with the nursing work, and it was worthy of promotion.

## 1. Introduction

Endoscopic retrograde cholangiopancreatography (ERCP) is a technique for X-ray cholangiopancreatography performed under the direct view of duodenoscopy by injecting human contrast agent through the duodenal papilla [1]. As a noninvasive examination and nonsurgical treatment, it is currently one of the important means for diagnosis and treatment of pancreatic and biliary diseases [2]. However, due to the lack of cognition about ERCP, patients generally present with negative emotions such as anxiety and tension, which will lead to hemodynamic changes and have a direct impact on the diagnosis and treatment of ERCP [3]. At the same time, under the influence of repeated intubation guidance, duodenal papilla sphincter dysfunction, angiography, and anesthesia and sedation drugs, most patients after ERCP have intestinal dysfunction, which affects the postoperative recovery [4]. The previous practice of ERCP has revealed that scientific and effective nursing intervention for patients is the key to ensure the safe and smooth implementation of ERCP.

Procedural nursing refers to a series of purposeful and planned nursing measures aiming at promoting the rapid recovery of patients, which can comprehensively and dynamically feedback the improvement of patients' function [5]. It has been used in the clinical care of patients with malignant tumor during the perioperative period, acute glomerulonephritis, coronary heart disease intervention, and other patients, and has received good feedback, but few studies have reported its application value in ERCP [6]. A thinking map belongs to a divergent visual thinking tool, which shows the boring relationship between different levels of topics with mutual membership and related hierarchy, and can provide users with clear path guidance and information support [7]. To improve hemodynamics and intestinal function of patients undergoing ERCP, a procedural nursing plan based on thinking map guidance mode was used in ERCP in this study, which is now reported as follows.

The article "Effect of Programmed Nursing Plan Based on Thinking Map Guidance Mode on Hemodynamics and Intestinal Function Recovery of Patients Undergoing Endoscopic Retrograde Cholangiopancreatography" was published in 2022. Journal: Emerg Med Int.

## 2. Materials and Methods

### 2.1. General Information

96 patients who received ERCP in our hospital from June 2019 to June 2021 were selected as research objects, which were divided into study group and control group according to the difference in nursing methods, with 48 patients in each group. This study has been approved by the medical ethics committee of the hospital, with the informed consent of patients or their families.

### 2.2. Inclusion Criteria

(1) Patients with clear indications of ERCP and undergoing ERCP [8]. (2) No history of mental illness. (3) Age ≥18 years.

### 2.3. Exclusion Criteria

(1) Patients with severe cardiopulmonary renal insufficiency. (2) Patients with autoimmune diseases. (3) Patients with systemic infectious diseases. (4) Patients with cognitive abnormalities. (5) Pregnant and lactating women.

## 3. Method

Patients in the control group received routine care. Before operation, the ERCP health education manual should be issued, and at the same time, patients should be given health education and routine psychological care. Before the examination, the routine blood test, urine amylase, and liver function of the patient were tested in accordance with the doctor's advice, and iodine allergy test and antibiotic allergy test were conducted, with antibiotics input intravenously. The contrast agent was prepared. The patient was instructed not to eat or drink for 6 h before the examination.

Patients in the study group were given routine nursing care in addition to that in the control group, and procedural nursing care based on thinking map guidance mode was also given.

1. An ERCP nursing group was formed and all members were organized to learn relevant knowledge such as ERCP, thinking map, and procedural nursing theory. With “ERCP care” as the central keyword, three Level 1 branches including preoperative nursing, intraoperative nursing, and postoperative nursing were diverged outward, into 11 Level 2 branches and eight Level 3 branches. A hierarchical structured thinking map for procedural care of patients undergoing ERCP was developed, as shown in Figure 1.
2. The nursing plan was orderly implemented according to the thinking map. (1) Preoperative care: to improve the preoperative preparation. At the same time, the patient data were analyzed, and preoperative health education and psychological care were targeted. Among them, health education was conducted in the form of multimedia education, in which patients were introduced to basic disease knowledge and ERCP knowledge, and informed to follow medical drugs, prevention of complications, follow-up examination, and other precautions. Psychological nursing takes psychological counseling, relaxation training, and social support as the main methods to relieve preoperative tension and anxiety of patients. (2) Intraoperative nursing: nursing staff should actively follow up the operating steps of the surgeons, strengthen cooperation with the surgeons, assist the surgeons to smoothly carry out the procedures of various operations, and speed up the process of surgery. During the operation, the monitoring of patients' basic vital signs such as pulse, consciousness, blood pressure, and oxyhemoglobin saturation was strengthened, and if any abnormality was found, the physician was informed immediately for treatment to prevent the occurrence of operation accidents. At the same time, after the contrast catheter was prepared, the intubation procedure was strictly followed, and the care for intubation was enhanced with professional skills. (3) Postoperative care: the patient's vital signs were closely monitored. We observed the symptoms such as abdominal pain, abdominal distension, and nausea and vomiting as well as yellow staining of the skin in our patient, and the traits, color, and volume of stool. If any abnormality occurred, we immediately informed the doctor to handle it. Always be alert to the occurrence of adverse events. Postoperative patients were assisted to carry out rehabilitation exercise as soon as possible to promote the recovery of gastrointestinal function. According to the needs of rehabilitation, the excessive care of patients from fasting to a low-fat liquid diet and then to a normal diet was strengthened to ensure nutritional support for patients. Psychological nursing was inserted in the process of nursing, in the same way as before the operation. Meanwhile, family members are required to provide emotional support, medication supervision, healthy life guidance, and complication prevention to ERCP patients.

The article "Effect of Programmed Nursing Plan Based on Thinking Map Guidance Mode on Hemodynamics and Intestinal Function Recovery of Patients Undergoing Endoscopic Retrograde Cholangiopancreatography" was published in 2022. Journal: Emerg Med Int.

### 3.1. Observation Indicators

1. The peripheral blood was collected at the time of admission (T0), before surgery (T1), at the end of the surgery (T2), and when awoke after surgery (T3). Three mL of blood was collected and centrifuged (1500r/min, 15 min) for separation and submission for examination. Mean arterial pressure (MAP) and heart rate (HR) were detected by chemical contrast staining.
2. The bowel sounds recovery time, postoperative anal exhaust recovery time, and postoperative first defecation time were compared between the two groups.
3. The self-rating anxiety scale (SAS) [9] and self-rating depression scale (SDS) [10] were used to assess the negative emotions of patients at the time of admission, before and after operation. The two tables contained 20 items, with each item scoring 1–4 points. The higher the score, the stronger the anxiety and depression were.
4. Comparison of the average hospitalization days, average medical cost, and satisfaction with nursing between the two groups was performed. Nursing satisfaction was recorded with the self-made nursing satisfaction questionnaire in our hospital. The full score of the scale was 100, with 90–100 being very satisfactory, 70–89 being satisfactory, 50–69 being general satisfactory, and <50 being unsatisfactory.
5. The incidences of hyperamylasemia, acute pancreatitis, acute cholangitis, diarrhea, and gastrointestinal hemorrhage in the two groups were counted.

### 3.2. Statistical Methods

All data were processed with the SPSS 22.0 statistical software, and GraphPad Prism 8 was used to make statistical graphs. The measurement data are expressed as mean ± standard deviation ($\bar{x}$ ± *s*), independent sample *t*-test is used for comparison between groups, count data are expressed as (n (%)), and the chi-square (*χ*^2^) test is performed. The difference is statistically significant when *P* < 0.05.

## 4. Results

### 4.1. Baseline Data

There was no significant difference in general data between the two groups, which was comparable (*P* > 0.05, Table 1).

### 4.2. Comparison of Hemodynamic Change between the Two Groups

Group (*F*_group_ = 36.43, 31.7103, *P*_group_=0.000) and time (*F*_time_ = 632.438, 20.628, *P*_time_=0.000) have an influence on MAP and HR, but there is no interaction between them (*F*_group_ _×_ _time_ = 1.563, 2.715, *P*_group× time_=0.199, 0.103, Table 2).

### 4.3. Comparison of Intestinal Function Recovery between the Two Groups

The bowel sounds recovery time, postoperative anal exhaust recovery time, and postoperative first defecation time were shorter in the study group than those in the control group (*t* = 12.687, 9.608, 5.004, *P* < 0.05, Figure.  2).

The article "Effect of Programmed Nursing Plan Based on Thinking Map Guidance Mode on Hemodynamics and Intestinal Function Recovery of Patients Undergoing Endoscopic Retrograde Cholangiopancreatography" was published in 2022. Journal: Emerg Med Int.

### 4.4. Comparison of Changes in SAS and SDS Scores between the Two Groups

Group (*F*_group_ = 12.223, 15.041, *P*_group_=0.001) and time (*F*_time_ = 264.825, 112.502, P_time_=) had an interaction on SAS and SDS scores (*F*_group_ _×_ _time_ = 7.837, 5.668, *P*_group×time_=0.006, 0.019, Table 3).

### 4.5. Comparison of the Average Hospitalization Days, Average Medical Cost, and Satisfaction with Nursing

Patients in the study group had shorter hospitalization days, less medical cost, and higher satisfaction scores than those in the control group (*P* < 0.05, Table 4).

### 4.6. Comparison of Complications between the Two Groups

The complication rate in the study group was lower than that in the control group (*P* < 0.05, Table 5).

## 5. Discussion

ERCP is an operationally challenging technique. Factors such as the patient's tolerance, the underlying condition, the anatomical structure, and the operator's empirical techniques all influence the successful and safe conduct of the procedure [11]. Therefore, it is very important to apply effective nursing methods to alleviate the stress response of ERCP patients.

The procedural nursing model is a new nursing model advocated in the field of clinical nursing at present, which was first proposed by Lott et al. [12]. Different from the traditional conventional care model, this model emphasizes that the surgical care process is divided into preoperative, intraoperative and postoperative parts, and each part is programmed to enhance the cooperation of nursing staff with the patients, families, and medical staff and improve the systematic and scientific nature of nursing [13]. Based on the research on previous literature, we found that the key point of procedural nursing was the nursing process, which could improve the effectiveness of nursing measures on the basis of formulating a scientific and effective nursing plan according to the priorities of clinical nursing work [14]. Thinking map is an effective graphical thinking tool to express divergent thinking [15]. It adopts the chart frame structure and compiles the complex and professional contents into a structure map with a high degree of organizational logic relationship [16]. The application of different lines to identify different hierarchical organizational structures can visually and clearly display the subordinate relationship among the theme of each hierarchy, which not only can ensure the identification and extraction of key information but also can avoid the omission of branch structure information. In clinical nursing, the hierarchical structure of “point with surface” in the thinking map was used to simplify information and highlight the focus of nursing work [17]. At the same time, the nursing measures were combined into a visual semantic network based on the internal correlation using tools such as words and images, to achieve the change from linear language logical thinking to space graphics with a clear hierarchical structure, which could make up for the deficiencies of language thinking, deepen the understanding of nursing staff, and improve work efficiency [18].

The article "Effect of Programmed Nursing Plan Based on Thinking Map Guidance Mode on Hemodynamics and Intestinal Function Recovery of Patients Undergoing Endoscopic Retrograde Cholangiopancreatography" was published in 2022. Journal: Emerg Med Int.

Since the gastrointestinal tract is distributed with rich autonomic nerve fibers, stimulation of the gastrointestinal tract by ERCP surgery will cause psychological and physiological stress responses of patients as well as hemodynamic abnormalities [19]. In addition, patients lack sufficient cognition and understanding of ERCP, and ERCP operation in a awake state easily aggravates emotional changes in patients [20]. Repeated measures in this study showed that group and time had effects on MAP, HR, and SAS and SDS scores, indicating that a procedural nursing plan based on thinking map guidance model could reduce the hemodynamic effects of ERCP on patients and alleviate their adverse psychology. Intestinal dysfunction after ERCP has also become a major clinical concern. At present, it is considered that the intestinal dysfunction caused by ERCP is related to the following factors: (1) Repeated intubation leads to papilledema and decreases in bile and pancreatic juice discharge [21]. (2) Dysfunction of duodenal papilla sphincter causes obstructed discharge of pancreatic fluid and bile as well as bile reflux. (3) Hemorrhage occurs after duodenal papilla incision [22]. (4) Influence of contrast examination and anesthetic sedative drugs. In this study, on the premise of assessing the patients' nursing needs, a scientific diet nursing plan was formulated according to the needs of postoperative gastrointestinal functional recovery, and on this basis, targeted, systematic, and effective nursing measures were implemented. The results showed that the bowel sounds recovery time, postoperative anal exhaust recovery time, and postoperative first defecation time were shorter in the study group than in the control group (*P* < 0.05). In addition, the incidence of complications in the study group was lower than that in the control group (*P* < 0.05). The reason was that in the nursing work of patients in the research group, through analyzing the patient's situation with the physicians, the nurses actively improved the preoperative preparation and effective nursing for complications, which not only improved the quality of surgery but also reduced the occurrence of complications [23].

In summary, the procedural nursing plan based on the thinking map guidance mode can reduce the hemodynamic effects of ERCP on patients, promote the recovery of intestinal function, alleviate their adverse psychology, reduce postoperative complications, help improve patients' satisfaction with the nursing work, and is worthy of promotion.

The article "Effect of Programmed Nursing Plan Based on Thinking Map Guidance Mode on Hemodynamics and Intestinal Function Recovery of Patients Undergoing Endoscopic Retrograde Cholangiopancreatography" was published in 2022. Journal: Emerg Med Int.

## Figures and Tables

**Figure 1:** Thinking map of procedural nursing care for patients with ERCP.

**Figure 2:** Histogram of comparison of intestinal function recovery between the two groups. Compared with the control group, ^*∗*^*P* < 0.05.

**Table 1:** Comparison of general data of patients between the two groups.

Group	n	Gender (n)		Age (years old)	Course of disease (months)	Type of disease (n)		Degree of education (n)		
		Male	Female			Biliary tract diseases	Pancreatic diseases	Junior high school or below	Senior high school or technical secondary school	College and above
Study group	48	26	22	46.25 ± 3.46	14.28 ± 3.17	29	19	12	16	20
Control group	48	25	23	46.59 ± 3.15	14.19 ± 3.52	30	18	14	15	19
*χ* ^*2*^/*t*	—	0.042		0.503	0.132	0.044			0.212	
*P* value	—	0.838		0.616	0.896	0.834			0.900	

**Table 2:** Comparison of hemodynamic changes between two groups ($\bar{x}$ ± *s*).

Group	n	MAP (mmHg)					HR (beats/min)		
		T0	T1	T2	T3	T0	T1	T2	T3
Study group	48	129.16 ± 5.83	104.31 ± 7.12	113.14 ± 4.20	95.11 ± 4.29	94.34 ± 8.35	80.96 ± 8.12	94.13 ± 4.25	82.83 ± 5.28
Control group	48	129.75 ± 5.64	106.26 ± 6.57	119.33 ± 5.29	99.48 ± 5.52	94.64 ± 8.71	86.65 ± 7.53	98.22 ± 3.24	87.17 ± 4.09

**Table 3:** Comparison of changes in SAS and SDS scores between the two groups ($\bar{x}$ ± *s*, score).

Group	*n*	SAS			SDS		
		On admission	Preoperatively	Postoperative	On admission	Preoperatively	Postoperative
Study group	48	50.39 ± 8.17	41.09 ± 5.13	32.26 ± 5.28	51.26 ± 7.52	43.33 ± 6.22	38.39 ± 5.84
Control group	48	50.46 ± 8.28	44.34 ± 6.10	36.19 ± 5.84	51.36 ± 7.57	48.34 ± 5.69	43.21 ± 5.78

**Table 4:** Comparison of the average hospitalization days, average medical cost, and satisfaction with nursing ($\bar{x}$ ± *s*).

Group	n	Average hospitalization days (d)	Average medical cost (million yuan)	Satisfaction with nursing (score)
Study group	48	7.22 ± 1.19	1.32 ± 0.16	94.28 ± 4.26
Control group	48	12.52 ± 2.63	1.79 ± 0.25	88.71 ± 5.93
*t*	—	12.720	10.971	5.258
*P* value	—	＜0.001	＜0.001	＜0.001

**Table 5:** Comparison of complications between the two groups (n (%)).

Group	n	Hyperamylasemia	Acute pancreatitis	Acute cholangitis	Diarrhea	Gastrointestinal hemorrhage	Total incidence
Study group	48	1 (2.08)	0 (0.00)	0 (0.00)	1 (2.08)	1 (2.08)	3 (6.25)
Control group	48	4 (8.33)	1 (2.08)	1 (2.08)	2 (4.17)	2 (4.17)	10 (20.83)
*χ* ^2^	—						4.360
*P* value	—						0.037

The article "Effect of Programmed Nursing Plan Based on Thinking Map Guidance Mode on Hemodynamics and Intestinal Function Recovery of Patients Undergoing Endoscopic Retrograde Cholangiopancreatography" was published in 2022. Journal: Emerg Med Int.

## Data Availability

For this test, relevant data are available upon reasonable request.
